# Changes in Physical Function of Shuttlecock Players after Short-Term Intensive Training based on Data Mining

**DOI:** 10.1155/2022/8153521

**Published:** 2022-06-13

**Authors:** Wenyao Zeng

**Affiliations:** College of Sport, Chongqing Technology and Business University, Chongqing 400067, China

## Abstract

This paper investigates the changes in body composition and physical fitness of badminton players after short-term high-intensity training. *Methods*. During an 8-week short-term training camp, 12 nonprofessional badminton players were paired to design training sessions, and body composition and fitness were measured before and after training. *Results*. After 8 weeks of high-intensity training, there was no significant change in body weight of badminton players (*P* > 0.05), while lean body mass increased significantly and body fat percentage decreased significantly (*P* < 0.05). The time of kicking, lying on the back, and standing forward was increased (*P* < 0.05), and the time of running back and forth 6.1 meters 3 times was shorter than that before training (*P* < 0.05). *Conclusion*. The increase of lean body mass can promote the energy conversion, oxygen consumption, and exercise capacity of athletes. Short-term training can reduce excess body fat, promote muscle development, and improve physical fitness.

## 1. Introduction

Shuttlecock, also known as kicking shuttlecock, has a long history and is popular. People who practice shuttlecock regularly can play better. Shuttlecock evolved from the Chinese shuttlecock sport and has an incredible and important position in traditional Chinese gymnasiums. Not only is it based on the sports, decoration, and fitness of badminton, but also it integrates badminton, volleyball rules, and football skills. Shuttlecock has become popular among people.

Shuttlecock was originally called “Net Shuttlecock,” which originated in Guangzhou and was officially renamed “Shuttlecock” after liberation. It has been developed in China for decades. In December 1928, when Shanghai held the “China Domestic Products Exhibition,” the shuttlecock competition was held for the first time, which promoted the development of the project. Since then, badminton competitions have been held across the country. In March 1933, Nanjing held the first national badminton competition, and a large number of badminton masters emerged. In October of the same year, Shuttlecock appeared in the National Games and made its first appearance in the comprehensive competition. In 1956, China held the first official badminton competition and formulated simple rules, marking the beginning of the badminton competition system. The promulgation of the “Rules of Shuttlecock Competition” in 1984 was an important turning point in Chinese shuttlecock regulation and a milestone in the history of Chinese shuttlecock development. At the same time, Shuttlecock was officially included in the sports competition items of the National Sports Commission. In April 1985, the former State Sports Commission held the first National Badminton Championships in Suzhou. In September 1987, the “China Badminton Association” was established in Beijing, and in the 5 individual competitions of the 5th World Badminton Championships held in Beijing, China, Chinese badminton players won all championships.

Shuttlecock is an ability developed by human beings that adapt and change naturally in daily life, study, work, and production habits. Shuttlecock is beneficial to chronic bone and joint diseases such as cervical spondylosis, shoulder and neck disease, lumbar disc herniation, and sciatica. It has a positive training effect on all aspects of the human body. The technical complexity of badminton varies from simple to difficult. It not only combines the physical and psychological characteristics of growth and development of problems with the regularity of human motor skills but also helps the growth and development of adolescents and improves the overall physical quality of adolescents. At the same time, badminton will be able to control the level and intensity of training during the training process, which will help train participants' aerobic endurance and improve their metabolism and blood supply to the heart. Participants regularly perform shuttlecock training, which can train each body's flexibility by capturing a three-dimensional sense of space and time, thereby improving physical coordination and flexibility. In addition, shuttlecock kicks are varied. You can compare the number of times, the time of consecutive kicks, and the pattern of kicks. Therefore, because of its simplicity, shuttlecock has become the first choice for the fitness of people of all ages.

## 2. Related Work

Xu et al. believe that the increasing popularity and development of data mining technology have brought a serious threat to the security of sensitive personal information. An emerging research topic in data mining, privacy-preserving data mining (PPDM), has been extensively studied in recent years. The basic idea of PPDM is to modify data in such a way that data mining algorithms can be executed efficiently without compromising the security of the sensitive information contained in the data. At present, the research on PPDM mainly focuses on how to reduce the privacy risk brought by data mining operations and realize data collection, data release, and information (i.e., data mining results) transmission [1]. Pearl et al. applied data mining techniques to discover relevant KPIs. This is a new method based on data mining to extract relevant KPIs [2]. Wang believes that shuttlecock is an excellent traditional national sport in China. Because of its simplicity, convenience, and fun, it is loved by the majority of people, especially teenagers and children. Before long, badminton has developed into a confrontational sport, and it takes a period of research to master badminton's tactics and strategies [3]. According to Chen et al., motion video analysis has been gaining popularity recently because of its importance in understanding motion and improving athlete performance [4]. According to Bourdon et al.'s monitoring, athlete load during training and competition has become a very hot topic in sports science. Both scientists and coaches often use a multidisciplinary approach to monitoring training loads, and the pursuit of the best way to capture and interpret data has led to an exponential growth in empirical and applied research. In fact, the field has grown so rapidly in recent years that it has spawned industries aimed at developing new styles that can precisely quantify an athlete's internal and external loads and help protect them from injury and disease [5]. Saw et al. believe that the athlete self-report measure (ASRM) has the potential to provide valuable insights into training response, but the disconnect between research and practice needs to be addressed. That is, the metrics or methods used in research do not always reflect practice, or the data obtained primarily from practice lack empirical quality [6]. Garthe and Maughan believe that, in elite sports, gestures are equal, and small factors can determine the outcome of sports competitions. Not all athletes know the value of making informed nutritional choices but anything that might give a competitive advantage, including dietary supplements. Supplements are typically used by 40% to 100% of athletes, depending on the type of sport, level of competition, and the definition of supplementation. However, unless the athlete is nutritionally deficient, supplementation may not improve performance and may adversely affect performance and health. Dietary supplements are classified as a subcategory of food, so manufacturers are not required to provide evidence of product safety and efficacy, nor do they need to obtain regulatory approval before selling supplements. This poses potential health risks, and serious adverse effects have been reported with the use of certain dietary supplements. Athletes participating in sports under antidoping regulations must also be aware that the use of supplements puts them at risk of ingesting prohibited substances or precursors of prohibited substances [7]. Brown et al. believe that precompetition screening is essential to rule out inherited heart conditions that can lead to sudden cardiac death in seemingly healthy athletes. Therefore, they considered whether a one-size-fits-all screening approach could account for individual differences in physical training, training volume, ethnicity, body size, gender, and age [8]. Bishop et al. found that strength- and jump-based tasks were most commonly used to examine these differences in the athlete and nonathlete populations. They examined the reliability, validity, and consideration of assessment to improve test accuracy and validity to quantify asymmetries in strength and jumping tasks [9]. In recent years, Thorpe RT has found that the increased demand for competition in elite team sports has prompted researchers and practitioners to place a strong emphasis on monitoring athletes' fitness and fatigue. Monitoring fatigue and understanding athlete status can also provide insights and useful information about athlete availability, injury, and disease risk. Traditional methods of quantifying recovery and fatigue in team sports, such as maximum fitness assessment, may not detect changes in fatigue status throughout the game. They faster, simpler, and nonexhaustive tests such as athlete self-report measurements and autonomic nervous system responses via heart rate derived indices. Robust rationalization and precise detection of meaningful fluctuations in these measures are critical for practitioners working with athletes and coaches daily [10].

## 3. Shuttlecock Training Method

Physical training can increase the physical fitness of athletes and is the basis of badminton. To compete, badminton players must undergo general physical training.

### 3.1. Speed Quality Training

Velocity quality refers to the ability of a human body to move quickly. It includes the ability of the human body to complete tasks quickly and respond quickly to external signal stimuli, as well as the ability to move quickly. In badminton, it is essential to improve the visual response ability of players. In the case of excitement, full of emotions, and strong desire to exercise, athletes should carry out quality training, which should generally be arranged in the first half of the training [11]. When the speed quality of a badminton player improves to a certain level, there are often stagnation and difficult progress. This is due to the formation of skill dynamic stereotypes, and the spatial and temporal characteristics of the athlete's technical movements tend to be stable. With the improvement of exercise level, athletes will encounter greater difficulties in improving the flexibility of nerve processes and the supply of energy required for muscle contraction, and the resistance that athletes need to overcome to move forward is also greater. At this time, you can use traction running, variable speed running, downhill running, leading running, and other methods to overcome.

### 3.2. Endurance Quality Training

Endurance quality refers to the body's ability to withstand long-term exercise. To maintain a specific exercise intensity or exercise quality throughout the game, badminton players must have good endurance qualities and be able to cope with the deep fatigue accumulated during continuous training. Improve endurance quality through cross-country running, long-distance running, ball sports, and so forth, improve the cardiopulmonary function of athletes, improve aerobic metabolism, and restore physical strength as soon as possible after high-intensity training. Therefore, badminton players should pay attention to endurance training, usually planning 1-2 hours of endurance training per week and planning more time for preparation and transition.

### 3.3. Strength Training

Strength quality refers to the ability of the human neuromuscular system to overcome or resist work stress. Shuttlecock requires the development of the upper and lower limbs, large and small muscles, and muscle groups, as well as the development of various joints and ligaments, especially the strength of the lower limbs. In the shuttlecock game, the offensive techniques commonly used by players in front of the net are dunk, turn dunk, and slap dunk. Therefore, it is necessary to exercise the strength of muscles and joints in different parts through different free exercises, including equipment, resistance, and boosting, while focusing on the strength of lower limbs, thighs, and abdomen, such as single-leg jumping, squat, half squat, stride, leapfrog, and skipping rope.

Comprehensive physical exercise can completely improve the basic quality of badminton players and improve their competitive level. However, the configuration should be reasonable, the methods should be more, and the monotony should be changed into active and interesting, which can effectively mobilize the enthusiasm of practice and enhance the effect of practice and do a good job of the special physical fitness training of shuttlecock players, so that they can further master the special sports technology and tactical level.

## 4. Data Mining and Research Methods

Data mining is a new business information processing technology. Its main feature is to extract, transform, analyze, and model a large amount of business data in business databases and extract key data to assist business decision-making. Relatively speaking, data mining has certain limitations, and its development and formation time is relatively short. Since its development in the 1990s, its application range has gradually expanded. It is not only beneficial to information processing but also of great significance to all aspects of production and life [12]. At this stage, data mining related technologies not only belong to the field of scientific research but also belong to the field of multidisciplinary technology. Therefore, data mining technology has been fully applied in all walks of life, and the technology is constantly improving and developing. Some scholars have come to a conclusion based on the actual situation that the meanings of modern information mining and data mining include the following:

1. Continuously enrich data on a real basis to realize massive data storage.
2. Use data mining, information collection, and value analysis to provide services for more industries, meet the data needs of different industries, and make life easier.
3. It is easier to be understood, accepted, and used by people, which can provide a basis for decision-making and can improve the scientific accuracy of decision-making through data analysis and judgment.

Data mining is generally related to computer science and achieves these goals through a number of methods such as statistics, online analytical processing, intelligence retrieval, machine learning, expert systems (relying on past rules of thumb), and pattern recognition [13].

### 4.1. Recording Method

This paper reviews the literature related to badminton and physical structure in the past 20 years as a theoretical basis. Through the library and CNKI retrieval of relevant materials, certain development status and characteristics have been found in the research on the physical structure of balls and badminton. This paper carefully reads and analyzes the obtained literature and data and obtains 45 original indicators of the body structure and characteristics of Chinese elite badminton players. The original test index data of the physical structure characteristics of Chinese elite badminton players is shown in Table 1:

### 4.2. Questionnaire Survey Method

Questionnaire refers to a form used in statistics and surveys to express questions in the way of asking questions. Questionnaire method is a method in which researchers use this kind of controlled measurement to measure the research questions, to collect reliable data.

This article takes advantage of the opportunity of many large and medium badminton matches in China to have extensive contacts and conversations with relevant experts and some coaches. On this basis, more than 50 cards were made, and the following factor set was established: the external performance factor set of badminton players' judgment ability. Although the athlete's judgment ability is an abstract concept, we can evaluate the athlete's judgment ability from six aspects through the external performance of the athlete in the game. The external performance factor set of badminton players' judgment ability is set as

(1) $$\begin{array}{c} U=\left\{u_{1},u_{2},u_{3},u_{4},u_{5},u_{6}\right\}. \end{array}$$

In the above formula, *u*_1_ is the purpose; *u*_2_ is the action; *u*_3_ is the predictability of the action; *u*_4_ is the agility of the action; *u*_5_ is the accuracy of handling the ball; it is the strain of handling the ball. *u*_6_ is the integrity of the fit.

Shuttlecock player training content factor set is as follows: We divide the training content usually implemented in training into 12 factors according to 6 categories: technique, tactics, body, psychology, competition, and summary. Let the training content factor set be as follows:

(2) $$\begin{array}{c} X=\left\{x_{1},x_{2},x_{3},\ldots ,u_{12}\right\}. \end{array}$$

In the above formula, *x*_1_ is research on rules and regulations; *x*_2_ is competition; *x*_3_ is regular technical training; *x*_4_ is irregular technical training; *x*_5_ is tactical knowledge learning; *x*_6_ is tactical routine practice; *x*_7_ is tactical awareness training; *x*_8_ is physical training; *x*_9_ is postmatch summary; *x*_10_ is watching games or videos; *x*_11_ is writing a training diary; *x*_12_ is cultural knowledge learning.

The questionnaire was compiled according to the factor set, and the method of questionnaire survey was adopted. Coaches and experts are required to judge the corresponding relationship between each training content factor in the questionnaire and the badminton player's judgment ability and set the relevant level to level 3. Fill in the form; fill in 1 if they think the two are similar; fill in 01 if they think the relationship is relatively close; fill in 0 if they think there is no relationship. Then, the data in all questionnaires were comprehensively sorted out, and the correlation coefficient between various training content factors and external performance was calculated. Finally, the correlation matrix *R* of *U* and *X* is obtained. In September 2005, taking advantage of the opportunity of the National Shuttlecock Championship held in Chengde City, Hebei Province, 100 questionnaires were distributed to coaches and related experts of 30 teams, where 90 questionnaires were returned, and 6 invalid questionnaires were excluded. The effective recovery was 84%.

### 4.3. Determination of Physical Fitness Indicators and Body Composition

Body fat is measured using the bioelectrical resistance method, which utilizes the principle of electrical resistance between adipose and nonadipose tissue. Conductors, muscles, and other stem cells have good electrical conductivity and high durability due to their high water content. Therefore, the proportion of fat and other substances can be measured by the electrical resistance of the body [14]. In the 15-second kick measurement, the subject used the attacking leg as the upper kick and the other leg as the supporting leg in a badminton match [15]. The number of kicks in 15 seconds is measured and tested with two heads: the subject lies flat on the mat with the arms straight, the shoulder blades must touch the mat, the knees are straight, and the head and hands are raised simultaneously. As much as possible, touch the toes as the person gets up and measure the number within a minute. In the 6.1 m back and forth 3 times, the test distance is a badminton court with a width of 6.1 m, and the subject runs from the starting point (side) to the end point (side). Touch the finish line with both hands, then touch the starting point, repeat 3 times, and sprint after touching the starting line. Perform 2 tests for the best record.

### 4.4. Features and Processes of Data Mining Technology

In the process of IoT data value extraction, key technical means show scalability and rotation capabilities, which can effectively utilize limited storage nodes and ensure data security [16]. Therefore, IoT stores data in different places based on the flow of data, each with its own unique classification. At the same time, IoT data is large and complex, which often requires a large number of sensor nodes, thereby improving the timeliness of processing important node information.

Processing data using statistical methods requires a series of processes. The data mining process is shown in Figure 1.

Data mining and cloud computing have become hot research fields today. Cloud computing is a type of distributed computing, which refers to decomposing large data computing processing programs into countless small programs through the network “cloud” and then processing and analyzing these small programs through a system composed of multiple servers to obtain results and return to the user. By building a distributed storage and distributed computing platform, data mining technology is used to process and analyze data. Cloud computing not only provides a powerful infrastructure for big data but also spawns a large number of big data processing technologies. The cloud service hierarchy is shown in Figure 2.

Cloud computing is the virtualization of hardware resources, and big data is the efficient processing of massive data. The schematic diagram of the data mining platform based on cloud computing is shown in Figure 3.

### 4.5. Cholesky Decomposition and Bayesian Models

Cholesky decomposition method, also known as square root method, is to express a symmetric positive definite matrix as a decomposition of the product of a lower triangular matrix *L* and its transpose.

To build the mathematical model, the coefficients are calculated. The model parameters *y* and *n* self-parameters *x*_*n*−1_,…, *x*_0_ must be randomly selected from the data samples, and the sorting and analysis of these parameters can be expressed by the following formula:

(3) $$\begin{array}{c} y=a_{0}x_{0}+a_{1}x_{1+\ldots +a_{n-1}x_{n-1}+a_{n}}. \end{array}$$

Bring these parameters into the formula for linear analysis, where the coefficient of the *a*_0_, *a*_1_,…, *a*_*n*−1_, *a*_*n*_ formula is a fixed value; according to the linear calculation rules of mathematics, the following must be calculated:

(4) $$\begin{array}{c} q=\sum_{i=0}^{m-1}{\left[y_{i}=\left(a_{0}x_{0}+a_{1}x_{1}+\cdots +a_{n-1}x_{n-1}+a_{n}\right)\right]}^{2}. \end{array}$$

The parameter coefficients *a*_0_, *a*_1_,…, *a*_*n*−1_, *a*_*n*_ must be able to fit the following system of linear formulas:

(5) $$\begin{array}{c} \left(CC^{T}\right)\left\{\begin{array}{c} \begin{array}{c} a_{0}\\ \begin{array}{c} a_{1}\\ a_{2} \end{array} \end{array}\\ \begin{array}{c} \begin{array}{c} \vdots \\ a_{n-1} \end{array}\\ a_{n} \end{array} \end{array}\right\}=C=\left\{\begin{array}{c} \begin{array}{c} y_{0}\\ \begin{array}{c} y_{1}\\ y_{2} \end{array} \end{array}\\ \begin{array}{c} \begin{array}{c} \vdots \\ y_{m-2} \end{array}\\ y_{m-1} \end{array} \end{array}\right\}, \end{array}$$

(6) $$\begin{array}{c} \text{Of which }C=\left[\begin{array}{ccc} \begin{array}{ccc} \begin{array}{c} x_{00}\\ x_{10}\\ \ldots \end{array} & \begin{array}{c} x_{01}\\ x_{11}\\ \ldots \end{array} & \begin{array}{c} x_{02}\\ x_{12}\\ \ldots \end{array} \end{array} & \begin{array}{c} \ldots \\ \ldots \\ \ldots \end{array} & \begin{array}{c} x_{0,m-1}\\ x_{1,m-1}\\ \ldots \end{array}\\ \begin{array}{ccc} x_{n-1,0} & x_{n-1,1} & x_{n-1,2} \end{array} & \ldots & x_{n-1,m-1}\\ \begin{array}{ccc} 1 & 1 & 1 \end{array} & \ldots & 1 \end{array}\right]. \end{array}$$

The calculation of Cholesky linear algebra can be decomposed as *A*=*U*^*T*^*U*, where *U* is a matrix, and the decomposition matrix is

(7) $$\begin{array}{c} \left[\begin{array}{ccc} \begin{array}{cc} \begin{array}{c} a_{00}\\ a_{10} \end{array} & \begin{array}{c} a_{01}\\ a_{11} \end{array} \end{array} & \begin{array}{c} \ldots \\ \ldots \end{array} & \begin{array}{c} a_{0,m-1}\\ a_{1,m-1} \end{array}\\ \begin{array}{cc} \ldots & \ldots \end{array} & \ldots & \ldots \\ \begin{array}{cc} a_{n-1,0} & a_{n-1,1} \end{array} & \ldots & a_{n-1,m-1} \end{array}\right]=\left[\begin{array}{ccc} \begin{array}{cc} \begin{array}{c} u_{00}\\ u_{10} \end{array} & \begin{array}{c} 0\\ u_{11} \end{array} \end{array} & \begin{array}{c} \ldots \\ \ldots \end{array} & \begin{array}{c} 0\\ 0 \end{array}\\ \begin{array}{cc} \ldots & \ldots \end{array} & \ldots & \ldots \\ \begin{array}{cc} u_{m-1,0} & u_{m-1,1} \end{array} & \ldots & u_{m-1,m-1} \end{array}\right]\times \left[\begin{array}{ccc} \begin{array}{cc} \begin{array}{c} u_{00}\\ 0 \end{array} & \begin{array}{c} u_{10}\\ u_{11} \end{array} \end{array} & \begin{array}{c} \ldots \\ \ldots \end{array} & \begin{array}{c} u_{0,m-1}\\ u_{1,m-1} \end{array}\\ \begin{array}{cc} 0 & 0 \end{array} & \ldots & \ldots \\ \begin{array}{cc} 0 & 0 \end{array} & \ldots & u_{m-1,m-1} \end{array}\right]. \end{array}$$

The factors of the *U* matrix are obtained by

(8) $$\begin{array}{c} U_{00}=\sqrt{a_{00}}, \end{array}$$

(9) $$\begin{array}{c} U_{ii}={\left(a_{ii-\sum_{k=0}^{i-1}u_{k}^{2}}\right)}^{1/2},\;i=1,2,\ldots ,m-1, \end{array}$$

(10) $$\begin{array}{c} U_{ij}=\left(a_{\left(ij-\overset{i-1}{\underset{k=0}{\sum }}u_{kiu_{kj}}\right)/u_{ij}}\right),\;j>i, \end{array}$$

and the formula *AX* = *B* can be given by

(11) $$\begin{array}{c} y_{i=\left(b_{i-\sum u_{kiy_{k}}}\right)/u_{ij}} \end{array}$$

(12) $$\begin{array}{c} x_{i=\left(y_{i-\overset{m-1}{\underset{k=i+1}{\sum }}u_{kix_{k}}}/u_{ij}\right)} \end{array}$$

The connecting line between two data samples of a Bayesian network is the mathematical relationship that exists between the data. Bayesian models are generally used in data analysis to solve problems such as prior probability, classification real-time prediction, and recommendation systems. Therefore, we introduce the classical Bayesian model:

(13) $$\begin{array}{c} P_{2}=\left\{X_{4},X_{5}\right\},\\ C_{2}=\left\{X_{1}\right\},\\ C_{4}=\left\{X_{2},X_{5}\right\},\\ P_{4}=\emptyset ,\\ P_{1}=\left\{X_{2},X_{3}\right\},\\ C_{1}=\emptyset . \end{array}$$

The Bayesian classical graph is shown in Figure 4.

The mathematical definition of the graph is the expression of the relationship between each data node in the model. This data model can be used to create a network graph and obtain the mathematical formula of joint probability:

(14) $$\begin{array}{c} P\left(X_{1}=x_{1},\ldots ,X_{m}=x_{m}\right)=\prod_{i=1}^{m}P\left(X_{i}=x_{i}|X_{j}=x_{j}\right). \end{array}$$

## 5. Analysis of Physical Function Changes of Shuttlecock Players

### 5.1. Questionnaire Survey Analysis

Using the correlation matrix method, the 84 collected questionnaires were divided into two equal parts, one of which was 42, and the rank values filled in each box were added up and then divided by 42, respectively. Correlation diagrams (Table 2 and Figures 5–7) are derived from this.

(15) $$\begin{array}{c} \text{R}=\left(r_{nm}\right)12\times 6\in \left[0,1\right], \end{array}$$

(16) rnm=nnpm=1×frequency+0.5×frequencyThe actual number of people who filled out the form.

Table 2 represents *x*_*i*_ (*i* = 1, 2, 3,…, 12) in *x*, that is, the degree of correlation between each training content factor and *U*, which specifies

(17) $$\begin{array}{c} A=\left\{a_{1},a_{2},a_{3},\ldots ,a_{m}\right\}, \end{array}$$

where

(18) $$\begin{array}{c} a_{m}=\overset{i}{\underset{m=1}{\sum }}r_{nm}j. \end{array}$$

The factor analysis of athletes' judgment ability and training content is shown in Table 2 and Figures 5–7.

The correlated changes in the values reveal the specific situation of the relationship between the training program factors and the badminton players' specific judgment ability for these 12 different types of badminton players. By analyzing the data in Table 2 and Figures 5–7, it can be seen that the data of the training items whose correlation coefficient is greater than 0.80 are arranged by size, and the coefficients are *X*_2_, *X*_7_, *X*_4_, and *X*_5_, respectively, as shown in Table 2, that is, in the badminton competition process, to cultivate badminton players' tactical awareness, irregular badminton sports technical training, and the use of tactics in competitions. It can be seen that the four training items have a great influence on the judgment ability of badminton players.

In this paper, the method existing in fuzzy mathematics is used to analyze and determine the relationship between badminton training items and badminton players' judgment ability. In this way, gathering originally scattered and vague viewpoints to form quantitative data can better help readers understand, grasp, and utilize the relationship between the two [17]. Through the analysis, it can be seen that the correlation between various training factors and badminton players' judgment ability is quite different. Therefore, badminton coaches can transform these factors into the main way to improve the judgment ability according to the actual situation of the players themselves.

### 5.2. Influence of Short-Term Intensive Training on Physical Function of Shuttlecock Players

Table 3 shows that, after 8 weeks of short-term training, the weight of badminton players did not change significantly (*P* > 0.05), and the lean body mass before training was significantly lower than that after training (*P* < 0.05). The body fat mass and body fat percentage before training were higher than those after training (*P* < 0.05). The body composition index data comparison of badminton players before and after training is shown in Table 3.

The total weight of the human body is made up of the various components of the human body. Excessive body fat may be detrimental to badminton players [18]. Excess fat is a burden on athletes, increasing their oxygen consumption and affecting their endurance, speed, and strength. This experiment found that, after 8 weeks of intensive training, the body fat content and body fat rate of badminton players were significantly lower than those before training. There was no difference in body weight before and after training. Because the training intensity, training time, and load are higher than normal training, most athletes engage in long-term aerobic exercise, which provides support for anaerobic exercise. Consumption of body fat by athletes results in a loss of body fat, a decrease in body fat percentage, and an increase in lean mass with little change in overall mass.

Lean body mass refers to the weight left after removing body fat. Muscle is an important part of lean body mass. During exercise, muscle is the driving force for athletes to work. A large number of studies have shown that lean body mass is closely related to the anaerobic energy of the human body. Oxygen capacity is highly correlated.

The data in Table 3 show that the fat-free body weight changed from 41.06 kg before exercise to 42.62 kg after exercise, with a large difference (*P* < 0.05), indicating that exercise has a muscle-building effect [19]. Lean body mass increases, the content of energy-supplying substances in muscle increases, and the ability of muscles to provide energy and metabolism during exercise also increases. Therefore, an increase in lean body mass can promote energy conversion, oxygen consumption, and exercise capacity in athletes.

### 5.3. Influence of Short-Term Intensive Training on Physical Fitness of Shuttlecock Players

It can be seen from Table 4 that, after 8 weeks of short-term training, the data of sitting posture, bending over, kicking, and lying on both sides after training are larger than those before training, and there is a big difference between the two periods (*P* < 0.05). The time-consuming reduction of the three 6.1-meter round-trip runs was significantly different from the pretraining data (*P* < 0.05). The comparison of physical fitness index data of badminton players before and after training is shown in Table 4.

From Table 4, it can be seen that the number of positive kicks in 15 seconds after training is more than that before training (*P* < 0.05), which reflects that the ability of athletes to quickly swing up and press down has been significantly improved. The number of people lying on the back for 1 minute after training was also more than that before training (*P* < 0.05), indicating that the strength and explosive power of the waist and abdominal muscles of the athletes were improved.

### 5.4. Discussion

Through 8 weeks of short-term physical fitness training and skill training, shuttlecock players have reduced body fat and increased lean body mass; muscle strength, flexibility, movement speed, and agility have been improved, and physical fitness and techniques and tactics have been fully developed.

The physical fitness of badminton consists of three parts: physical fitness, body shape, and physiological function. All elements restrict and promote each other. Changes in any element will affect the development of the overall physical fitness of the athlete.  Figure 8 shows the body structure of Chinese elite badminton players.

To establish the ideal body structure model of Chinese elite badminton players, teaching and research personnel need to determine the evaluation indicators, calculate the eigenvalues of the indicators, determine the weights of the indicators in the physical fitness indicator system, and conduct repeated revisions and tests. By connecting each independent link, this paper finally constructs an ideal physical structure model workflow, as shown in Figure 9.

## 6. Conclusion

There is a close relationship between badminton players' psychological, physical, technical, and other factors. For example, physical fitness is a prerequisite for skills, but physical fitness is relatively more susceptible to innate traits, and skills can be continuously developed. Therefore, through a lot of research, this paper finds out the influence of various factors on badminton players' judgment ability and then draws a conclusion. Most badminton players should focus more on improving their ability to judge factors such as technique and tactics, which can be greatly improved [20]. It is hoped that the concepts and conclusions obtained in this paper can help Chinese badminton players to quickly improve their judgment ability and then achieve better results in the competition. The research on the physical function changes of shuttlecock players after short-term intensive training based on data mining is also of great significance for promoting the development of current shuttlecock players.

## Figures and Tables

**Figure 1:** Data mining flow chart.

**Figure 2:** Cloud service hierarchy.

**Figure 3:** Cloud computing-based data mining platform.

**Figure 4:** Bayesian classical graph.

**Figure 5:** Athletes' judgment ability and training content factor 1.

**Figure 6:** Athletes' judgment ability and training content factor 2.

**Figure 7:** Athletes' judgment ability and training content factor 3.

**Figure 8:** Physical fitness system diagram of Chinese elite badminton players.

**Figure 9:** Flow chart of the construction of the physical fitness model of Chinese elite badminton players.

**Table 1:** The original test indicators of the body structure characteristics of Chinese elite badminton players.

Serial number	Test indicators	Serial number	Test indicators	Serial number	Test indicators
1	High	16	Leg length and height	31	30 meters (seconds)
2	Sitting height	17	Achilles tendon length/calf length	32	4-second run (m)
3	Upper limb length	18	Quotation index	33	Plate
4	Leg length	19	Lung capacity	34	Standing long jump
5	Achilles tendon length	20	VO2 max	35	Squat barbell
6	Calf length	21	30 squats in 30 seconds	36	Vertical jump in place
7	Shoulder width	22	Resting heart rate	37	Crunches (60 s)
8	Hip width	23	Postexercise pulse	38	Push-ups
9	Foot width	24	Blood urea	39	10 m round trip (4*∗*100 m)
10	Waistline	25	Body fat percentage	40	5 : 30 move
11	Hip circumference	26	Lean body mass	41	800 meters
12	Thigh circumference	27	5 meters	42	12-minute run
13	Calf circumference	28	Stroop test	43	Seated forward bend
14	Ankle	29	One-minute dribble	44	Cross
15	Weight	30	One-minute stomp	45	Longitudinal fork

**Table 2:** Correlation matrix between athletes' judgment ability and training content factors (*r*_*nm*_).

	*u*_1_	*u*_2_	*u*_3_	*u*_4_	*u*_5_	*u*_6_	A sort of
*x*_1_	0.41	0.45	0.46	0.26	0.42	0.40	0.41
*x*_2_	0.96	0.95	0.84	0.87	0.94	0.95	0.92
*x*_3_	0.70	0.55	0.62	0.75	0.80	0.59	0.66
*x*_4_	0.78	0.84	0.78	0.70	0.82	0.87	0.81
*x*_5_	0.85	0.86	0.80	0.81	0.78	0.62	0.80
*x*_6_	0.90	0.73	0.66	0.69	0.82	0.71	0.75
*x*_7_	0.93	0.87	0.85	0.78	0.83	0.79	0.84
*x*_8_	0.40	0.27	0.76	0.48	0.19	0.45	0.42
*x*_9_	0.85	0.63	0.52	0.50	0.69	0.62	0.63
*x*_10_	0.92	0.61	0.42	0.58	0.84	0.77	0.69
*x*_11_	0.80	0.47	0.53	0.59	0.50	0.41	0.55
*x*_12_	0.55	0.44	0.19	0.34	0.18	0.38	0.35

**Table 3:** Comparison of body composition indexes of badminton players before and after training.

Grouping	Weight (kg)	Lean body mass (kg)	Body fat (kg)	Body fat percentage (%)
Before training	51.9 ± 1.43	40.06 ± 2.47	7.40 ± 0.15	15.53 ± 2.22
In training	51.7 ± 0.91	40.93 ± 1.83	6.97 ± 0.11	15.12 ± 2.89
After training	51.4 ± 0.66^*∗*^	41.62 ± 1.44^*∗*^	6.42 ± 0.07^*∗*^	14.80 ± 3.17^*∗*^

*Note.* Comparison before and after training: ^*∗*^*P* < 0.05.

**Table 4:** Comparison of physical fitness indicators of badminton players before and after training.

Grouping	Kick (individual/15 s)	Supine (person/min)	Standing forward bend (cm)	6.1 m 3-round trip (s)
Before training	16.89 ± 1.93	18.22 ± 6.39	15.56 ± 5.60	9.93 ± 0.66
In training	17.51 ± 2.23	22.13 ± 5.15	16.31 ± 5.10	9.64 ± 0.51
After training	18.33 ± 2.57^*∗*^	25.44 ± 5.69^*∗*^	17.78 ± 4.74^*∗*^	9.30 ± 0.56^*∗*^

*Note.* Comparison before and after training: ^*∗*^*P* < 0.05.

## Data Availability

Data sharing is not applicable to this article as no datasets were generated or analyzed during this study.
